The article "Evaluating Evidences of Effectiveness in Web-Based Nursing Education Program" was retracted in 2023. Reasons: unreliable results or conclusions; concerns about the data; concerns about the peer review; concerns about the citations.

# Evaluating Evidences of Effectiveness in Web-Based Nursing Education Program

**DOI:** 10.1155/2021/3901916

**Published:** 2021-11-25

**Authors:** Jie Wang

**Affiliations:** Bengbu Medical College, China

## Abstract

**Background:**

Web-based education programs are essential in every field of learning, and in nursing coursework, they can contribute towards behavioral development. It is found that emerging approach of web-based nursing programs is overpowering the traditional education methods and provides flexibility in learning and training programs. Therefore, it is considered as a promising medium of learning which can take over the traditional methods because of its effectiveness.

**Objective:**

A systematic review and meta-analysis was performed for analysis of efficiency and effectiveness of web-based nursing education. This study is aimed at evaluating the evidences which evaluate the effectiveness of the web-based nursing education programs. *Material and Methods*. Studies were selected from 2008 to 2020 available from various global databases like PubMed, Embase, CINAHL, ProQuest, and Cochrane Library.

**Results:**

Five studies were selected for analysis where the results demonstrated no significant difference in the effectiveness of use of web-based nursing educational programs.

**Conclusion:**

More evidences are required for supporting the efficiency and effectiveness of use of web-based programs for nursing education. Hence, more research is required for evaluating the length of nursing education, evaluating practice-based clinical aspects like success ratio for outcomes of study, type of patients handled, and severity of cases handled for better outcomes.

## 1. Introduction

Many research studies describe that the duration spend by the students in class diminishes the timeline in the clinical placements and eventually in the process of learning practical expertise [1]. The procurement of these clinical abilities is important for the undergraduate nursing program. The unsuitable education and unfavorable clinical abilities balance the excellence of care and safety assured to the patients [2]. The nurse instructors experience the problems of accommodating and assessing the teaching procedures in order to train nurses for upcoming transformations in the healthcare sector.

Each of these methods used in teaching is utilized in the coursework of nursing, and it should benefit the high-level learning programs, the real-time implementation, and critical analysis skills. The productive proposal to analyze the teaching skills and methods in the coursework nursing program are not properly defined in the literature. The ingenious teaching skills and activities utilized by the nursing tutors are rarely analyzed. The discipline of web-based nursing education programs has accumulated consideration in the literature in the recent times. The experts have suggested for employing evidence-based online teaching methods (EBTs) and have recognized proficiency for the nursing tutors [3].

The verification needed to counsel and analyze the web-based teaching methods in the nursing programs still lacks the clarity [4]. These nursing tutors might be accustomed with the evidence-based online teaching methods but not much familiar with the evidence-based approaches needed to analyze their teaching skills and methods. The advancement of nursing programs to the web-based or mobile-based platforms is the expansion of teaching methods which is favored by the technical evolution of the computing devices, which paves a way to the web-based learning is the demand of the present flexible society [5].

The evidence-based approaches are resolution-oriented strategies towards clinical care which integrates the diligence usage of the present suitable evidence from a well-structured study, clinician's skills, and the preferences raised by the patients [6, 7]. However, the evidence-based programs have developed to a substantial limit in the past few years and are a crucial notion by the healthcare experts. The integration of these programs is still under the process and remains a challenge in the nursing sector as well the accumulation of the evidence-based practice in application, and the web-based nursing programs still remain a crucial affair.

The progress made by the developed nations is higher in the accumulation of the evidence-based practice in the routine of patient care as well as the training process of the healthcare experts. Although the evidence-based practice remains in the onset when it comes to the developing nations, however such countries have obvious benefits for the productive utilization of the healthcare and related resources. The development of evidence-based practices in online nursing programs needs to obtain the proficiencies in the areas like literacy of knowledge about informatics, statistics, and research methodology to issue an essential premise for additional knowledge. Thus, raising the evidence-based practice seldom obtains the outstanding outcomes within the short-term continuation of the nursing-based education program [8].

According to McKimm [9], the fundamental attributes of a web-based nursing program can be listed as follows: (a) the coursework, notices, and the time-table structure; (b) the study material like the presentations and handouts; (c) the curriculum framework; (d) discussion sessions and establishing communication via email; (e) regular assessment activities; (f) student management programs like tracking performance, records, and marksheets; and (g) referring to the available online library, database, and articles. Additionally, the mode of teleconference [10], case study-based learning methods [11], and the online credit-oriented coursework [12] are some crucial procedures used in the web-based nursing education programs.

## 2. Method

### 2.1. Search Strategy

The electronic database available in English was identified for the search strategy that falls in the period of 2003 to 2021, available from PubMed, Embase, ProQuest, and Cochrane Library. The investigation was done following the guidelines presented by the PRISMA (Preferred Reporting Items for Systematic Reviews and Meta-Analysis).

### 2.2. Inclusion and Exclusion Criteria

A total of 179 research studies were identified applicable to this study using the search MeSH terms: “e-learning,” “web-based learning,” “online learning,” “online nursing program,” “nursing education,” “case-based learning,” “web-based education,” “computer learning,” “nursing,” “nursing student,” and “randomized allocation or randomized controlled” utilizing clinical databases and other databases. Apart from these studies, additional 4 databases were also included as per the inclusion criteria. Out of all these identified studies, only 92 were shortlisted as relevant as per the study and 91 were found to be duplicate records. The screened 92 studies were further reviewed, and only 5 of them were identified relevant as per the aim of this study, where 87 were rejected as per the exclusion criteria. The rejected articles were as follows: not available in English, had unclear outcomes, only abstracts, review paper, inapplicable study designs, selective reporting, and missing conclusions. The PRISMA used for selection of studies is shown in Figure 1, and characteristics of studies are shown in Table 1.

St. mean Diff for 95% CI is 0.29 (-0.03-0.61) with heterogeneity *I*^2^ = 71% (CI: confidence interval). Forest plot on effect of population size selected for the web-based programs for nursing courses on their knowledge is shown in Figure 2, and funnel plot for the same is in Figure 3.

St. mean difference with 95% CI is 0.47 (0.23-0.70) with high heterogeneity as *I*^2^ = 88% (CI: confidence interval). Forest plot on analysis of the role of blended knowledge on web-based education in nursing is shown in Figure 4 and funnel plot on Figure 5.

St. mean difference with 95% CI is 0.59 (0.33-0.85) with low heterogeneity as *I*^2^ = 0% (CI: confidence interval). Forest plot on analysis of web-based education on clinical performances in nursing is shown in Figure 6 and funnel plot on Figure 7.

St. mean difference with 95% CI is 0.17 (-0.07-0.41) with very low heterogeneity as *I*^2^ = 1% (CI: confidence interval). Forest plot on analysis on the role of program type web-based knowledge on web-based education in nursing is shown in Figure 8 and funnel plot on Figure 9.

St. mean difference with 95% CI is 0.52 (0.25-0.78) with very low heterogeneity *I*^2^ = 88% (CI: confidence interval). Forest plot on analysis of 4-week time on knowledge and its effect on web-based nursing education program is shown in Figure 10 and funnel plot on Figure 11.

St. mean difference is 0.35 (-0.02-0.72) with heterogeneity of *I*^2^ = 74% (CI: confidence interval). Forest plot on analysis of the web-based education program on nursing students on their knowledge is shown in Figure 12 and funnel plot on Figure 13.

## 3. Discussion

We conducted a study for evaluation of effectiveness of e-learning/web-based nursing programs for nursing students or professionals. On using random effect models, we have found that there is no significant difference noted on clinical performance/learner's knowledge. Though some studies suggest that a collaborative use of traditional and web-based learning will be useful, we did not find any such significant results. Hence, these programs are useful for those who cannot enroll in a traditional education environment.

Subgroup analysis of web-based knowledge as the program type and blended knowledge program type for web-based education showed no significant difference in the effects. The standard mean and the effect size had no significant effects.

Further analysis was performed on the participant type which were nursing students and the effect of web-based education program on their knowledge. No significant differences in the effect size were noted; hence, it was concluded that nursing profession requires in-depth training to imbibe clinical skills via experimental practical training which cannot be restricted to online or web-based mode.

Analysis of the 4-week intervention time for training resulted in no significant difference in the effect size, thereby concluding that the duration of intervention has no effect as receiving and learning time spent by the nursing students/practitioners cannot determine the effect size unless accurate time spent on each course is mentioned precisely.

The meta-analysis we performed for evaluation of the web-based nursing education programs has limitations of the difference in variables in the studies. Thus, characteristics were variable.

The efficiency and quality of web-based nursing program when compared with traditional methods are enlisted in this study. Some limitations like adult respiratory nursing care with clinical skill variation are not listed. Though blended learning methods will be effective for new learners, a longer duration of implementation of e-learning has to be done.

## 4. Conclusion

The study provided a better insight on the understanding of web-based education program for nursing students, researchers, and professions. The results were nonsignificant; hence, web-based nursing programs may contribute if assessed for longer period of times. Hence, in future meta-analysis, it might be possible to further evaluate the scope of this study by adding more variables like self-efficacy, parameters of clinical standards, self-satisfaction, and clinical outcomes.

## Figures and Tables

**Figure 1:** PRISMA study for the learning process.

**Figure 2:** Forest plot on effect of population size selected for the web-based programs for nursing courses on their knowledge.

**Figure 3:** Funnel plot of population size on nursing courses based on their knowledge.

**Figure 4:** Forest plot on analysis on the role of blended knowledge source program type on web-based education in nursing.

**Figure 5:** Funnel plot on the effect of blended knowledge program on web-based education.

**Figure 6:** Forest plot on analysis of web-based education on clinical performances in nursing.

**Figure 7:** Funnel plot on effect of web-based education on their clinical performances.

**Figure 8:** Forest plot on analysis on the role of program type (web-based knowledge) on web-based education in nursing.

**Figure 9:** Funnel plot on effect of (web-based knowledge) program type on web-based nursing education.

**Figure 10:** Forest plot analysis of 4-week time on knowledge and its effect on web-based nursing education program.

**Figure 11:** Funnel plot on the effect of intervention time on knowledge due to web-based education program.

**Figure 12:** Forest plot on analysis of the web-based education program on nursing students on their knowledge.

**Figure 13:** Funnel plot on web-based education program on nursing students on their knowledge.

**Table 1:** Description of studies.

Characteristics					
Author	Choi [13]	Lu et al. [14]	Kim et al. [15]	Joshi et al. [16]	Hwang et al. [17]
Country	Korea	Australia	Korea	India	Korea
Participants	Nurses	Student nurses	Nurses	Student nurses	Student nurses
Study design	Nonrandomized clinical trial	N/A	Nonrandomized clinical trial	Randomized controlled trial	Quasi-experimental, pretest-posttest design
Year of study	2012	2009	2011	2013	2012
Intervention duration	4 weeks	N/A	4 weeks	N/A	8 weeks
Measures of outcome	Web-based learning	Blended web-based learning	Blended web-based learning	Web-based learning	Web-based learning

## Data Availability

The data used to support the findings of this study are available from the author upon request.
